The article "Antitumor Molecular Mechanism of Chlorogenic Acid on Inducting Genes GSK-3β and APC and Inhibiting Gene β-Catenin" was retracted in 2021. Reasons: no approval from a third party; copyright claims.

# Antitumor Molecular Mechanism of Chlorogenic Acid on Inducting Genes GSK-3****β**** and APC and Inhibiting Gene ****β****-Catenin

**DOI:** 10.1155/2013/951319

**Published:** 2013-06-16

**Authors:** Ruoshi Xu, Qiumei Kang, Jie Ren, Zukun Li, Xiaoping Xu

**Affiliations:** ^1^West China School of Stomatology, Sichuan University, Chengdu, Sichuan 610041, China; ^2^West China School of Pharmacy, Sichuan University, Chengdu, Sichuan 610041, China

## Abstract

*Objective.* Inhibiting gene **β**-catenin and inducting genes GSK-3**β** and APC, promoting the tumor cell apoptosis in Wnt pathway, by chlorogenic acid were discussed (CGA). *Method.* The different genes were scanned by the 4∗44K mouse microarray chips. The effect of the three genes was confirmed by RT-PCR technique with CGA dosage of 5, 10, and 20 mg/kg. *Result.* The expression of GSK-3**β** and APC was upregulated in group of 20 mg/kg dosage (*P* < 0.05) and the expression of **β**-catenin was downregulated in the same dosage (*P* < 0.05). *Conclusion.* The results infer that the multimeric protein complex of **β**-catenin could be increased by CGA upregulated genes GSK-3**β** and APC, which could inhibit the free **β**-catenin into the nucleus to connect with TCF. So the transcriptional expression of the target genes will be cut to abnormal cell proliferation. It is probably one of the ways that can stop the tumor increase by CGA.

## 1. Introduction

Chlorogenic acid is the ester of caffeic acid and quinic acid in shikimate pathway, which is commonly found in some plants, such as honeysuckle, Cortex Eucommiae, Semen Coffea Arabica, and green tea. Chlorogenic acid has antibacterial, antiviral, clear free radicals, and antitumor effects [1]. In recent years, the effective anticancer activity and low toxicity of chlorogenic acid were constantly confirmed and draw the attention of the people [2–4]. Kurata et al. [5] showed that the inhibition of tumor cell proliferation effect of chlorogenic acid was enhanced with increasing dose; they speculated that this inhibition of tumor cell proliferation may be obtained by enhancing the activity of the DNA ladder and caspase-3 as well as increasing the expression of c-Jun. Gmnado and Feng et al. showed that the in vitro experiments show that the anticancer mechanism of CGA contains inhibition of cell growth, regulation of cell cycle, and induction of apoptosis pathways, such as (1) to reduce ROS expression to reduce cell growth/reproduction signal transduction pathway of NF-*κ*B, AP-l, and MAPKs to reduce cancer cell viability, (2) to improve the activity of the NAD (P)H and GST, (3) to inhibit the expression of tetradecanoyl method wave alcohol acetate (TPA), in order to reduce the c-Jun NH2-terminal kinase, p38 kinase, and MAPK kinase-4 to prevent cancer transformation, and (4) to stimulate the expression of NF-E2-related factor and the activity of GST regulated by Nrf2 downstream cascade links antioxidant response element (ARE) to inhibit the growth of cancer cells [6, 7]. Chlorogenic acid is considered to be an effective cancer chemical repellant because of its significant inhibitory effect on colorectal cancer, liver cancer, and laryngeal [8]. In this paper, the biological gene chip technology was used to detect the variation of a whole set of gene sequences in breast tumor-bearing mice cells in the dynamic treatment cycle with CGA. The differential genes were screened by using genomics profiling, which was also the potential target gene associated with tumor disease according to the gene GO characteristic quality. Further verification testing must be designed, such as accurate quantitative PCR technology and western blot technology, to verify the potential target point in the treatment of chlorogenic acid for tumors. 

## 2. Instrument and Material

### 2.1. Tumor Lines and Animals

 EMT-6 mice breast tumor lines were preserved by Key Laboratory of Transplant Engineering and Immunology, Ministry of Health, West China Hospital, Sichuan University. Female BALB/C mice, weighing 17~18 g, and originally purchased from Experimental Animal Center of Sichuan University, have been bred in the ordinary small animal housing of the same center where the feeding conditions comply with GB 14925-2001 with the ambient temperature of 19 ± 3°C and humidity of 55 ± 15%. 

### 2.2. Instruments and Regents

CO_2_ incubator (MCO-15AC, SANYO, JP), biological safety cabinets (NU-425, NUAIRE, USA), electronic balance (JY12001, Sartorius, USA), high-speed centrifuge (TGL-16G, Shanghai, China), PCR (ABI-9700, ABI, USA), hybridization oven (G2545A, Agilent, USA), scanner (G2565BA, Agilent, USA), spectrophotometer (ND1000, NanoDrop, Autoclave), Quantitative PCR instrument (Bio-Rad, USA), IQ2-cryogenic high-speed centrifuge, standard 96-well plate, Clean Bench, Sujing Group Aetna, ChemiDoc XRS + system medium (Gibco, China), Calf serum (Minhai, Lanzhou, China), 0.25% trypsin (Gibco, USA), double antibiotics (penicillin and streptomycin sulfate) (North China), Cy3 NHS ester (lot no. PA13105), GE healthcare, aaUTP Ambion (AM8436), Low RNA Input Linear Amplification Kit (lot no. 5184–3523), Gene Expression Hybridization Kit (lot no. 5188–5242), 5188–5327 Gene Expression Wash Buffer Kit (including wash buffers 1 and 2), Stabilization and Drying Solution (lot no. 5185–5979), Gasket slide (lot no. G2534-60003a), 4*44K mouse microarray, Hybridization CGAmber (lot no. G2534A), Agilent USA, RNeasy Mini kit (lot no. 74106), QIAGEN, USA. Trizol reagent, Invitrogen. DEPC, Oligo, 5x reaction buffer, Riblock Rnase Inhibitor, dNTP MIX, RevertAid M-MulV, 2*Taq Master Mix novoprotein, IQTM SYBR Green Supermix, Bio Rad. RevertAid First Strand cDNA Synthesis Kit, Fermentas, fluorescent imager DNA ladder, novoprotein, chlorogenic acid for injection (CGA, lot no. 061101, 30 mg), white powder for injection (content of 99.87%), offered by Sichuan Jiuzhang Biological Chemical Technology Development Co. Ltd. Docetaxel for injection (DX, lot no. 10112611, 20 mg), purchased from Jiangsu Hengrui Medicine Co. Ltd. IFN*α*-2b (20110908, 500 IU) purchased from Anhui Anke Biotechnology (Group) Co. Ltd. 0.9% saline (NS, lot no. A060418) (Kelun, Sichuan, China).

### 2.3. Preparation of Sample Solution

To use CGA solution, CGA freeze-dried powder was dissolved with sterile saline to make concentrations of CGA sample solution that were 1, 0.5, and 0.25 mg·mL^−1^, respectively.

To use DX solution, 20 mg of DX injection powder was diluted with 1.5 mL of special solvent. To this, about 8.0 mL of saline was added to be stock solution of 2 mg·mL^−1^. The stock solution was diluted to be sample solution with the concentration of 0.25 mg·mL^−1^ with saline before use.

To use IFN*α*-2b solution, IFN*α*-2b was diluted with 20 mL sterilized saline. 

## 3. Methods

### 3.1. Preparation of Balb/c-EMT-6 Mice Model

#### 3.1.1. Preparation and Subcultivation

The anabiotic EMT-6 breast tumor lines were implanted subcutaneously into the right forelimb of mice. The tumor-bearing mice were obtained until the tumor grew to 1 cm × 1 cm × 1 cm. Then took out the tumor, cleaned it with NS, weighed it, cut it into pieces, and placed it in a homogenizer. NS (about 1 : 4) was added to the homogenizer, and cell suspension was obtained after fast homogenate. 0.2 mL of the cell suspension was inoculated subcutaneously into the right forelimb of mice and was randomized.

#### 3.1.2. Experiment Design

30 female BABL/C mice were randomly divided into 6 groups (*n* = 5), including normal saline (negative) group, CGA high-dose group (20 mg·Kg^−1^), CGA middle-dose group (10 mg·Kg^−1^), CGA low-dose group (5 mg·Kg^−1^), DX positive control group (5 mg·Kg^−1^), and IFN*α*-2b positive control group (5 million U·Kg^−1^). 

After being inoculated for 24 hours, the NS group, CGA groups, and IFN*α*-2b positive control group were continuously subcutaneously administered for 12 days. The DX group was administered interday for 6 times. The tumors were taken after 24 hrs of the last administration, then weighed, cut into pieces, frozen in liquid nitrogen, and stored at −70°C after segmentation package.

### 3.2. Detection of the Level Changes of Cell Gene with Gene Chip

#### 3.2.1. Total RNA Extraction

The lysis/binding buffer was added, 1 mL per 0.1 g tissue, for homogenate on ice to prevent RNA degradation. Adding homogenate additive (1/10) into the homogenate; the homogenate was vortexed, mixed, and kept on ice for 10 min. Then added phenol and chloroform mixture in the same volume as lysis, vortex them for 30 s, centrifuged them in 10,000 g for 5 minutes at room temperature. Added the absolute ethanol to the supernatant, then vortex and mixed them, made them going through the purification column repeatedly, centrifuged them at 10000 g for 15 seconds, discarded the supernatant. Added 350 *μ*L Wash I, centrifuged them for 5 s to purify the column, then centrifuged at 10,000 g for 15 s, discarded filtrate. Added 10 *μ*L DNase I and 70 *μ*L buffer RDD to the film, placed them for 15 min, and then successively added 350 *μ*L Wash 1 and 500 *μ*L Wash 2, centrifuged them for 5 s, cleaned the purification columns two times. Each cleaning must be centrifugal at 10,000 g for 15 s and discard the filtrate. Added 100 *μ*L 95°C preheated nuclease-free water to spin column and placed the spin column in a new collection tube after the second cleaning. The total RNA would be obtained after centrifuging at the maximum speed for 30 s and then stored at −70°C.

#### 3.2.2. Purification of Total RNA

QIAGEN RNeasy Kit was used for further extraction and purification of the total RNA. 100 *μ*L RNase-free water was added to dissolve the total RNA, then mixed with 350 *μ*L buffer RLT and 250 *μ*L ethanol. (The preparation of RLT: 14 mL original RLT can be added to 140 *μ*L of *β*-mercaptoethanol.) Transferred the sample to the RNeasy column, centrifuged at 10000 g for 30 s, and abandoned filtrate. Clean the RNeasy minicolumn twice with 500 *μ*L buffer RPE, centrifuged at 10,000 g for 30 s and 2 min, respectively, and discard the filtrate. Add 40 *μ*L RNase free water to the column, and centrifuge 10000 g for 1 min. Repeat the operation once more; the purified RNA was prepared.

#### 3.2.3. Total RNA Quality Testing

The quality of total RNA can be determined with agarose gel electrophoresis. Prepare the electrophoresis buffer 50x TAE, which was processed with DECP and autoclaves → a 1% agarose gel was prepared after adding on amount of agarose to lx TAE electrophoresis buffer → run on a gel for 15 min, then observe and picture the gel over the gel imager → lab-on-chip.

### 3.3. Validation of Protein Expression of Specific Genes by Fluorescence Quantitative PCR

#### 3.3.1. Primers and Reaction Conditions

The primers were designed through the 01190 software and synthesized by Sangon Biotech (Shanghai). The primer information of these four genes was shown in Table 1. With the template of sample cDNA, the differentially expressed genes were verified to use SYBR Green by real-time fluorescent quantitative PCR. The conditions of the q-PCR reactions were subjected to 94°C for 10 min, followed by 40 cycles at 94°C for 15 s and 54.5°C for 30 s, and finally 72°C for 45 s. The expression levels of GSK-3*β*, APC, and *β*-catenin in test samples were detected with GAPDH as the reference gene and calculated by 2^−ΔΔCT^ relative quantification method, which showed the differential expression of different groups compared to the NS group.

#### 3.3.2. RNA Extraction

After isinfecting the reagent bottle, boxes, and gloves under UV light for 30 min, the tissues were homogenized in the trizol reagent. The homogenate was incubated at 15–30°C for 5 min, to which chloroform was added, then vortex them for 15 s, and centrifuged separating the mixture for 15 min in low temperature. Transferred the upper supernatant into another tube, added 0.5 mL isopropanol and mixed them at 15–30°C, incubated them for 10 min, 4°C, then centrifuged them at 12000 g for 10 min, discarded supernatant, and added 1 mL 75% ethanol into the tube, centrifuged them at 7500 g for 5 min, discarded the supernatant, and dried them in the air for 3−5 min. Added 20 *μ*L DEPC deionized water to dissolve the RNA and stored them at −70°C.

#### 3.3.3. RNA Quality Testing

(1) *OD Value Detection.* A260/A280 value was determined by UV with 1 *μ*L extracted from each of RNA which was diluted to 100 *μ*L with TE buffer. 

(2) *RNA Formaldehyde Electrophoresis.* The voltage of conditions electrophoresis was 80 V, and running time was 40 min. The RNA samples prepared in Section 3.3.2 were diluted with DEPC water suitably and mixed with an equal volume of sample buffer, then heated for 4 min in boiling water, cooled on ice for 2 min, and then centrifuged in 1200 rpm for 5 s. The sample was spotted on plate to be carried on the electrophoresis.

#### 3.3.4. The Synthesis of cDNA

The RevertAid First Strand cDNA Synthesis Kit was used for reverse transcription. The total reaction volumes of RT-PCR reactions were 20 *μ*L. The system consists of 2 *μ*L RNA, 1 *μ*L Oligo(dT)18 primer, 9 *μ*L RNase-free water, 4 *μ*L 5x reaction buffer, 1 *μ*L Riblock Rnase Inhibitor, 2 *μ*L 10 mM dNTP MIX, and 1 *μ*L RevertAid M-MulV. 

The reverse transcription system liquids of the above were subjected to 42°C, 60 min, and 70°C, 5 min, in a PCR instrument. The reaction products were stored at −80°C for long-term preservation.

#### 3.3.5. The Test of RT-PCR Amplification Products

Briefly, the presence or absence of the only bands was observed at 496 bp as the standard showed the quality of cDNA. If there is one and only one band, the PCR product cDNA was qualified, and Q-PCR can be the next. The voltage was 130V, and the analysis time was 25 min.

The RT-PCR amplification system had 25 *μ*L liquid of total reaction volumes, in which consists of 10 *μ*L 2x Taq Master Mix, 2 *μ*L cDNA, 0.75 *μ*L Forward GAPDH primer pair and 0.75 *μ*L Reverse GAPDH primer, and 11.5 *μ*L RNase-free water. PCR reactions were subjected to 94°C for 10 min, followed by 40 cycles at 94°C for 15 s and 54.5°C for 30 s and finally 72°C for 45 s.

#### 3.3.6. Real-Time Fluorescent Quantitative PCR

1 *μ*L cDNA was diluted to 100 *μ*L with sterile water on standby. Gene primers, F and R, were diluted 20-fold, respectively. This reaction system was shown in Table 2. Each sample should go through the three parallel tests, taking the mean value to calculation. 

#### 3.3.7. SYBR Green I Reaction Designed and Optimized

(1) *Optimization of the Annealing Temperature.* By setting a certain temperature range, we can screen the optimal annealing temperature by real-time quantitative PCR reactions. The melting curve can be used to assess the specificity of the reaction in the quantitative PCR instrument. If there are multiple peaks on the melting curve, which indicates nonspecific products such as primer dimer, they are amplified along with specific products simultaneously, which also indicates the primers of the reaction need to be redesigned.

(2) *Construction of the Standard Curve.* cDNA was selected as the template and set eight 10-fold dilution series of points each dilution was repeated three times. The equation of the linear regression line has obtained the logarithmic value of template initial concentration as the abscissa and the CT value as the vertical coordinate. Standard curve correlation coefficient (*r*) or the coefficient of determination (*R* ^2^) can be used to evaluate the degree of linearization with the specific requirements of *r* > 0.990 and *R* ^2^ > 0.980.

## 4. Results

### 4.1. Results of CGA Suppression of the Mice Breast Cancer (EMT-6)

See Table 3.

### 4.2. Electrophoresis Graph and Lab-on-Chip

As is shown in Figure 1, the luminance ratios of 28 s and 18 s are greater than or equal to 2 in electrophoresis graph, which preliminary determines that total RNA was qualified. The result has shown that the quality of RNA extracted from each group of tumor tissue samples meets the requirement of further detection of gene chip. Then the differential genes closely related to the tumor cell suppression in the course of treatment were screened by the time series analysis, GO analysis, and pathway analysis and validated with q-PCR.

### 4.3. The Quality Results of RNA, cDNA

(1) *The Results of OD Values.* As is shown in Table 4, the A260/A280 value of RNA was from 1.63 to 2.18, which meets the quality requirements of RNA. 

(2) *Formaldehyde Electrophoresis of RNA.* As is shown in Figure 4, the formaldehyde denaturing electrophoresis showing the 28S and 18S were clear without DNA impurity band and degradation RNA, which meets the requirements of the experiment.

(3) *Results of cDNA Quality Test.* As is shown in Figure 5, there is only one band at 496 bp, which indicates that the quality of the PCR product meets the requirements.

### 4.4. PCR Expression of GSK-3*β*, APC, and *β*-Catenin

The PCR expression of GSK-3*β*, APC, and *β*-catenin was shown in Figure 6 in the tumor tissue of Balc-b/EMT-6 tumor-bearing mice after the treatment of DX (5 mg/kg), IFN (5 × 10^6^ U·kg-1), CGA (20 mg/kg), CGA (10 mg/kg), and CGA (5 mg/kg) for 12 days. Compared with the blank group, the expression of GSK-3*β* and APC was upregulated in group of 20 mg/kg dosage (*P* < 0.05) and the expression of *β*-catenin was downregulated in the same dosage group (*P* < 0.05).

## 5. Discussion

(1) As shown in Table 3, compared to the positive control group of cytotoxic anticancer drugs DX, biological response modifier (BRM) IFN groups, and the negative group of NS, the three dosag of the CGA groups showed better antitumor effect (*P* < 0.05); especially the inhibition rate of the 20 mg·kg^−1^dose group was more than 50%, which was equivalent to 59.92% of the DX group and 40.80% of the IFN group. It is suggested that chlorogenic acid should be able to be a new good anticancer agent in future clinical application.

(2) According to the data of the different time points in the inhibitory process acquired with the total RNA that was qualified in Figures 1, 2, and 3 the differential genes closely related to the Wnt pathway in the course of treatment were screened by the time series, GO, and pathway. The different genes which were connected with CGA treatment were extracted and were confirmed with q-PCR. The downward trends of the tumor genomes 18 and 21 were screened by the logarithm of standardization and fitting the change course of genes with similar trends; the genetic trend was closer to the fitted values of *P* smaller, such as Figures 7(a) and 7(b).

(3) As shown in Figure 7(a), the trend of genome 18 was confirmed to the anticancer process of CGA. According to the analysis of KEGG signaling pathway and the characteristics of GO in genome 18, some downregulated genes were found which are related to the tumor suppression pathway, such as BdnF mediated MAPK, Cflar, Cln3 Ddit3 Notch2 Rps6, Sox9, Spn, and Ppp1r13l. The gene 21 time sequence diagram relates to the Wnt pathway, mTOR pathway, the Notch pathway, and some immune-related pathways, such as B cell receptor pathway, T-cell receptor pathway, and metabolic pathway. It was inferred that CGA had a multipathway to inhibit the tumor growing up.

(4) Because our animal model was a breast cancer (EMT-6/BALB-C), we focused on the influence of Wnt pathway (shown in Figure 8) which was a special pathway that the breast cancer had. In particular, the gene glycogen synthase kinase 3(GSK-3*β*) and downstream gene ubiquitin ligase E3(APC) were upregulated. And the two kinds of genes had closed relationship, in which the gene APC was upregulated by upstream gene GSK-3*β*. And then, both genes could cause the down-stream gene *β*-catenin to downregulate directly in the Wnt pathway. As you know, the cancer will be developing when the gene *β*-catenin expression was upregulated. What is the gene *β*-catenin? From its GO searching revealed, *β*-catenin is a multifunctional protein, which can assist the cells react to extracellular signal and changes by interaction with the cytoskeleton. This protein acts as a transcription (transcription) factor in the nucleus to promote cell division genes. The accumulation of *β*-catenin would lead to abnormal activation of the downstream transcription factors after transferring to the nucleus, which mainly cause tumor. So, it is suggested that the *β*-catenin inhibited was one of the ways to inhibit tumor growth. On the other hand, the upregulation of GSK-3*β* is a multifunctional serine/threonine class of protein kinase, which plays an important role in the Wnt/wingless, PI3-kinase, and Hedgehog signaling pathway with the physiological functions including transcriptional activation, cell proliferation, and cell differentiation, cell movement. It can phosphorylate shaft protein and *β*-catenin, cause the degradation of *β*-catenin protein, and thereby inhibit the activation of the pathway. The activated APC plays an important role in promoting complexes degradation in a fast, efficient, and highly selective way in the anaphase cell cycle, which also can phosphorylate shaft protein and *β*-catenin, cause the degradation of *β*-catenin protein, and thereby inhibit the activation of the pathway. So the activation of GSK-3*β* and APC and downregulation of *β*-catenin in the group of CGA suggested that CGA could inhibit tumor by activating GSK-3*β* and APC.

(5) As shown in Figure 6(a), the regulation confirmed by Q-PCR in treatment process of CGA for EMT-6 breast cancer indicates groups of CGA in each dose and DX can activate expression of GSK-3*β*, especially the CGA 20 mg/kg group and the DX group can significantly upregulate GSK-3*β* (*P* < 0.05). As shown in Figure 6(b), groups of CGA at 20 mg/kg and 10 mg/kg and DX can activate expression of APC, but groups of CGA at 5 mg/kg dose little to upregulation. As shown in Figure 6(c), DX group, IFN group and CGA 20 mg/kg group was inhibited gene *β*-catenin.

## 6. Conclusion

 It is suggested that affecting the gene expression of GSK-3*β*, APC, and *β*-catenin by chlorogenic acid in Wnt pathway was one of the targets in the multipathway to antitumor of CGA.

## Figures and Tables

**Figure 1:** The EC of CGA 1–4.

**Figure 2:** The EC of CGA 5-6, DX, and blank.

**Figure 3:** The EC of DX3 and blank.

**Figure 4:** RNA electrophoresis.

**Figure 5:** cDNA electrophoresis.

**Figure 6:** The average PCR expression of different genes in different groups. (a) GSK-3*β*, (b) gene APC, and (c) gene *β*-catenin.

**Figure 7:** The expression trend graphs of gene 18 and gene 21 (*P* = 0).

**Figure 8:** Wnt signaling pathway.

**Table 1:** The Primer information of these four genes.

Gene symbol	Forward primer	Reverse primer
GSK-3*β*	ACC ATC CTT ATC CCT CCA	CAg Aag Cgg CgT TAT Tg
APC	CAC TgA gAA TAA ggC TgA C	TTC CgT AAT ATC CCA CC
*β*-Catenin	ggT gCT ATT CCA CgA CT	CCC TTC TAC TAT CTC CTC C
GAPDH	CAA GGT CAT CCA TGA CAA CTT TG	GTC CAC CAC CCT GTT GCT GTA G

**Table 2:** The reaction system of q-PCR (*n* = 3).

Composition	Plus the amount
IQ SYBR Green Supermix	10 *μ*L
Forward primer	1 *μ*L
Reverse primer	1 *μ*L
cDNA	2 *μ*L
Nase-free water	6 *μ*L

Total volume	20 *μ*L

**Table 3:** Results of CGA suppression of the mice breast cancer.

Groups	Dose (mg·kg^−1^)	Animals	Average tumor weight (g)	The average tumor inhibition rate (%)
DX	5	5	0.780 ± 0.244**	59.92
IFN	5 million U·kg^−1^	5	1.152 ± 0.254**	40.80
CGA	5	5	1.326 ± 0.254**	31.86
CGA	10	5	1.222 ± 0.363**	37.20
CGA	20	5	0.968 ± 0.633**	50.26
Negative	—	5	1.946 ± 0.233	—

**Table 4:** OD value of RNA.

No.	Group 1	Group 2	Group 3	Group 4	Group 5	Group 6
1	1.86	2.08	2.18	2.07	2.18	2.15
2	1.95	2.09	2.17	2.09	2.04	2.16
3	2.05	2.12	2.23	2.09	1.90	2.17
4	1.63	2.07	2.14	2.10	1.94	2.19
5	2.15	2.06	2.18	2.13	1.95	2.17
